# Protocatechualdehyde Inhibits the Osteoclast Differentiation of RAW264.7 and BMM Cells by Regulating NF-*κ*B and MAPK Activity

**DOI:** 10.1155/2021/6108999

**Published:** 2021-07-16

**Authors:** Yunyun Qu, Xin Liu, Shuai Zong, Huanxin Sun, Shuang Liu, Yueran Zhao

**Affiliations:** ^1^Department of Central Lab, Shandong Provincial Hospital, Cheeloo College of Medicine, Shandong University, Jinan, Shandong 250021, China; ^2^The Second Affiliated Hospital of Shandong University of Traditional Chinese Medicine, Jinan, China

## Abstract

Protocatechualdehyde (PCA), an important component of *Salvia miltiorrhiza*, has many activities, such as anti-inflammatory and antisepsis activities. However, the role of PCA in osteoclasts is not clear. We used RAW264.7 cells (a mouse leukemic monocyte/macrophage cell line) and bone marrow macrophages (BMMs) to probe the role of PCA in osteoclasts and the underlying mechanism. The effects of PCA on cell activity were evaluated with CCK-8 assays. TRAP staining detected mature osteoclasts. Corning Osteo Assay Surface plates were used to examine absorption. The levels of RNA and protein were analyzed, respectively, using RT-PCR and Western blotting. PCA (5 *μ*g/ml) was not toxic to the two cell types but reduced the formation of osteoclasts and bone absorption. Furthermore, PCA restrained the expression of mRNAs encoding proteins associated with osteoclasts and reduced the phosphorylation of proteins in important signaling pathways. The results indicate that PCA inhibits osteoclast differentiation by suppressing NF-*κ*B and MAPK activity.

## 1. Introduction

Osteoporosis is a degenerative disease with an increasing risk due to aging and is one of the most common diseases in older men [1]. The disease can occur at any age but mainly occurs in elderly men. Approximately 200 million people suffer from osteoporosis worldwide, and this condition has become the seventh most common disease in the world.

Under normal circumstances, bone tissue maintains normal function by constantly updating metabolism. Due to abnormal metabolism, older patients experience bone loss. The increased activity of osteoclasts increases the loss of bone mass, and the attenuated function of osteoblasts decreases the formation of bone mass, leading to fractures in the bone microstructure and a negative balance in bone reconstruction [2]. Therefore, more bone loss than supplementation is the cytological basis for the occurrence of osteoporosis.

Currently, bisphosphonates are common agents used to treat osteoporosis and significantly inhibit the activity of osteoclasts. They have been recommended by many authoritative institutions worldwide due to their clear efficacy [3]. However, the safety of long-term bisphosphonate use has gradually become a concern. Long-term application of bisphosphonates was reported to cause mandibular osteonecrosis, atypical subtrochanteric or femoral shaft fracture, and other adverse reactions [4].

*Salvia miltiorrhiza* (SM) is a Chinese herbal medicine that has long been used to treat osteoporosis. Clinical trials have shown that SM alone is as effective as traditional drugs in the treatment of osteoporosis and has the advantage of being nontoxic [5]. *In vitro* experiments have confirmed that SM exerts a good protective effect on ovariectomy-induced osteoporosis and diabetic osteoporosis [6, 7]. Salvianolic acid B is a water-soluble extract of SM. It exerts a protective effect on prednisone-induced osteoporosis [8], increasing bone cancellation, improving the bone trabecular structure, and increasing bone density.

Protocatechualdehyde (PCA) is the main degradation product of salvianolic acid B and has many activities, such as anti-inflammatory and antibacterial properties [9]. *In vivo*, the prodrug PCA restrains the destruction of the femoral condylar cartilage caused by adjuvant arthritis [10]. PCA significantly improves bone physical indexes, increases bone density and the levels of bone minerals and organic matter, increases the ratio of important organs, and effectively prevents the occurrence of osteoporosis caused by prednisone acetate in the growth period of rats [11]. However, the role of PCA in osteoclasts is not clear.

In this study, RAW264.7 cells (a mouse leukemic monocyte/macrophage cell line) and bone marrow macrophages (BMMs) were used to analyze the role of PCA in osteoclasts and the underlying mechanism. PCA has important theoretical significance and clinical application value in the search for economical and effective drug monomers to treat osteoporosis.

## 2. Materials and Methods

### 2.1. Materials

RAW264.7 cells were selected from ATCC (Manassas, VA, USA). BALB/c mice were purchased from Shandong University. PCA (purity > 98% by HPLC) was obtained from Sigma. Cell culture media were obtained from BI. Cytostimulators were acquired from R&D Systems. CCK-8 and TRAP kits were purchased from Sigma. 24-well bone plates were purchased from Corning Life Science (Lowell, MA, USA). Phalloidin was obtained from Thermo Fisher Scientific. The apoptosis kit was purchased from BD. All antibodies were acquired from Cell Signaling Technology (Beverly, MA, USA). Primers were designed by PrimerBank and synthesized by Shanghai Bioengineering Company.

### 2.2. Cell Culture

BMMs were acquired from both ends of cut femurs and tibias from approximately 6-week-old male BALB/c mice. The animal experiment was authorized by the Experimental Animal Ethics Review Committee of Shandong University. The marrow cavity was rinsed 3-5 times with *α*-MEM, and red blood cells were removed to obtain BMMs. The lysate was filtered through a 40 *μ*m mesh filter and centrifuged to separate the cells. Samples from the mice were cultured overnight in *α*-MEM containing M-CSF (5 ng/ml) in a nonadherent culture plate, and then, cells suspended in the collected supernatant were cultured with M-CSF (30 ng/ml) for 3 days. The supernatant and suspended cells were discarded; the adherent cells were the BMMs.

RAW264.7 cells were cultured in complete DMEM. However, DMEM was substituted for *α*-MEM to culture osteoclasts induced by receptor activator of nuclear factor-*κ*B ligand (RANKL).

### 2.3. Cytotoxicity Assay

CCK-8 assays were used to determine the toxicity of PCA toward cells. In 96-well plates, BMMs (2 × 10^4^ cells/well) and RAW264.7 cells (1 × 10^4^ cells/well) were seeded in the presence of PCA (0, 1, 10, 20, 30, or 50 *μ*g/ml) for 5–6 days. CCK-8 (10 *μ*l/well) was added to the supernatant and incubated for 0.5–1 h, and the absorbance was assayed at 452 nm by a Multiskan Go1510 microplate reader. The ratio of the experimental group to the control group represents cell activity [12].

### 2.4. TRAP Staining

RAW264.7 cells (5 × 10^3^ cells/well) were cultured in 48-well plates, and BMMs (2 × 10^4^ cells/well) were seeded in 96-well plates. The next day, 50 ng/ml RANKL and 30 ng/ml M-CSF were added to the BMM culture media, and 50 ng/ml RANKL was added to the RAW264.7 culture media. In addition, PCA (0, 1, 2.5, or 5 *μ*g/ml) were added to the medium. After 4–6 days, the cells were stained and identified according to the literature [13].

### 2.5. Absorption Pit Assay

We used Corning Osteo Assay Surface 24-well plates to assay absorption pits. BMMs (4 × 10^5^ cells/well) and RAW264.7 cells (1 × 10^5^ cells/well) were seeded and incubated for 24 h. Next, 50 ng/ml RANKL and 30 ng/ml M-CSF were added to the BMM culture media, and 50 ng/ml RANKL was added to the RAW264.7 culture media. In addition, PCA (1, 2.5, or 5 *μ*g/ml) was added at the same time, and the cells were incubated for 4–8 days. After 4–8 days, a 10% bleach solution was used to wash the cells. A light microscope (Olympus) captured images of the absorption pits, and ImageJ software quantified the image [14].

### 2.6. Immunofluorescence Staining of the F-Actin Ring

BMMs (3 × 10^5^ cells/well) were seeded in 24-well plates, and a series of PCA, M-CSF (30 ng/ml), and RANKL (50 ng/ml) were added to the medium. The cells were incubated for 4 days, and phalloidin was used to stain the cells after fixation and permeabilization. A fluorescence microscope was used to capture fluorescence images.

### 2.7. Flow Cytometry Analysis

RAW264.7 cells (5 × 10^5^ cells/well) were seeded in 6-well plates and cultured with a series of PCA and 50 ng/ml RANKL. After 3–4 days, the apoptosis kit was used to stain the cells. Cell apoptosis was assessed using flow cytometry.

### 2.8. RT-qPCR

RAW264.7 cells were seeded in 24-well plates (5 × 10^4^ cells/well). The next day, the cells were pretreated with a series of PCA concentrations for 60 min before adding 50 ng/ml RANKL. After 5–6 days, the cells were collected. PCR was performed as previously described [15]. Primers were listed in Table 1.

### 2.9. Western Blot Analysis

RAW264.7 cells (2.5 × 10^6^ cells/m) were plated in 6-well plates and then pretreated with PCA (1, 2.5, or 5 *μ*g/ml) for 2 h before the addition of RANKL (50 ng/ml) and incubation for 10 min. Western blots were performed as previously described [11]. The levels of p-p38/p38, p-ERK/ERK, p-JNK/JNK, and p-p65/p65 are shown in histograms.

### 2.10. Statistical Analysis

The results are presented as means ± standard errors. Each experiment was repeated more than three times. SPSS19.0 software was used to analyze differences. *P* < 0.05 was defined as a statistically significant difference.

## 3. Results

### 3.1. PCA Attenuates Osteoclast Differentiation Induced by RANKL

The potential cytotoxicity of PCA toward RAW264.7 cells (Figure 1(a)) and BMMs (Figure 1(b)) was evaluated using CCK-8 assays. Based on the results, the highest concentration of PCA (5 *μ*g/ml) has no effect on cell activity.

BMMs and RAW264.7 cells were successfully induced to differentiate into osteoclasts by RANKL. The osteoclasts were large and full, with vacuoles forming in the middle and additional nuclear accumulation throughout the cells. However, when PCA was present, the size of the osteoclasts decreased, the vacuoles disappeared, and the number of surrounding nuclei decreased. Furthermore, we used TRAP to stain osteoclasts. The test results indicated that PCA prevented osteoclastic differentiation not only in BMMs but also in RAW264.7 cells (Figures 1(c)–1(f)). Thus, PCA attenuates the generation of osteoclasts.

We added 5 *μ*g/ml PCA to the medium and induced BMMs to differentiate in three periods to determine the stage of osteoclastogenesis at which PCA exerted its effect. Osteoclast formation was markedly inhibited by PCA in the earlier period (Figures 1(g) and 1(h)), whereas the inhibitory effect of PCA decreased in the later period. These data suggested that PCA suppresses osteoclast formation mainly in the earlier period of RANKL-induced differentiation.

### 3.2. PCA Decreases the RANKL-Induced Formation of Absorption Pits

The absorption of osteoclasts induced by RANKL was detected. The group stimulated with RANKL formed obvious bone absorption pits, but the number and area of absorption pits decreased in the presence of PCA (Figure 2). Therefore, PCA inhibits the function of osteoclasts.

### 3.3. PCA Suppresses the Size of F-Actin Rings and Does Not Affect Apoptosis

The size of the F-actin ring was measured, and PCA reduced the length of the F-actin rings (Figures 3(a) and 3(b)). However, the flow cytometry analysis showed that PCA did not affect the ratio of apoptotic cells (Figures 3(c) and 3(d)). These data suggested that the inhibitory effect of PCA is not attributable to apoptosis.

### 3.4. PCA Attenuates the mRNA Expression of RANKL-Induced Osteoclastic Markers

The RT-qPCR results showed the mRNA levels of factors produced by RANKL-stimulated osteoclasts. The RANKL-induced group exhibited substantially increased expression of these mRNAs (Figure 4). However, PCA significantly reduced the mRNA levels of these related factors.

### 3.5. PCA Suppresses the Activation of the MAPK Pathway

The MAPK signaling pathway exerts an irreplaceable effect on the generation of osteoclasts. Primary members of this signaling pathway are ERK, JNK, and p38. Phosphorylation of these proteins is the main indicator of activation. We measured the levels of these proteins produced during the formation of osteoclasts in cells treated with or without PCA. The RANKL-induced group exhibited substantially increased phosphorylation of these proteins. However, the changes were inhibited by PCA (Figure 5).

### 3.6. PCA Prevents RANKL-Induced NF-*κ*B Activation

The change in p65 expression was examined. We measured the levels of p65 phosphorylation during RANKL-stimulated differentiation of cells treated with or without PCA. As shown in Figure 6, the RANKL-stimulated group exhibited increased p65 phosphorylation. However, when PCA was present, the level of p65 phosphorylation was decreased. These results indicate that PCA prevents NF-*κ*B activation induced by RANKL.

## 4. Discussion

Osteoclasts are derived from promonocytes in bone marrow hematopoietic stem cells and are mainly present in the periosteum. Osteoclasts are the only cells with bone absorption functions, initiating the process of bone remodeling and clearing old bone matrix [16]. Therefore, decreasing osteoclast differentiation or absorption may be an effective method to treat this type of pathological bone disease. This study was the first to show that PCA significantly inhibited the formation and function of RANKL-induced osteoclasts. In addition, PCA effectively inhibited the expression of osteoclast-associated marker genes stimulated by RANKL. Mechanistically, PCA suppressed RANKL-induced activation of the MAPK and NF-*κ*B signaling pathways.

We used two types of osteoclast progenitors (BMMs and RAW264.7 cells) to study the roles of PCA in the induction and absorption function of osteoclasts [17]. Through the research, we discovered that RAW264.7 cells only proliferated in the absence of stimulation, and the proliferation of BMMs only gradually decreased. However, when stimulated with RANKL, these cells all differentiated into osteoclasts and showed absorption functions. This result is consistent with the literature [13, 14]. Furthermore, this effect was inhibited by PCA. These actions were neither related to the cytotoxic effects of PCA nor a cause of apoptosis. Therefore, we further examined the mechanism of PCA in osteoclasts.

A series of iconic factors are produced in the course of differentiation from precursor cells to mature osteoclasts and thus can be used as markers of osteoclasts and their differentiation stages. Cathepsin K (CTSK) is an amino acid protease expressed by osteoclasts. CTSK stimulates the expression of TRAP on osteoclasts *in vitro*; thus, CTSK is an important factor for determining osteoclast function [18]. The recombinant nuclear factor of activated T-cells, cytoplasmic 1(NFATc1) is the most important factor associated with NF-*κ*B in the incipient stage of osteoclast formation. *In vitro* experiments confirmed that stem cells lacking NFATc1 fail to differentiate into osteoclasts, but ectopic NFATc1 expression in the absence of RANKL also enables BMMs to differentiate into osteoclasts [19]. These results all suggest the importance of NFATc1. Matrix metalloproteinase (MMP-9), which is abundant in osteoclasts, is an important protease that stimulates bone absorption. Specifically, MMP-9 plays a crucial function in the active transcription of osteoclastogenic genes via the cleavage of the N-terminal tail of H3 under tight epigenetic regulation [20]. Dendritic cell-specific transmembrane protein (DC-STAMP), an important molecule involved in the fusion of mononuclear cells into osteoclasts, improves the absorption function of osteoclasts [21]. Cellular oncogene FOS (C-FOS) is a protooncogene associated with the development of osteosarcoma. During osteoclast differentiation, C-FOS is an indispensable downstream regulatory factor of RANKL, which accelerates the formation of osteoclasts by activating the downstream factor NFATc1 [22]. In the present study, PCA reduced the mRNA levels of these factors. Therefore, PCA may inhibit the formation of osteoclasts by downregulating the expression of these genes. However, these genes are downstream of the signaling pathway, and the mechanism by which PCA modulates these downstream genes remains unclear. Therefore, we detected the levels of proteins in the MAPK and NF-*κ*B signaling pathways.

MAPK is an important signaling pathway involved in osteoclast differentiation [23]. This pathway mainly activates and regulates key downstream regulatory molecules associated with the formation of osteoclasts, including C-FOS and NFATc1 [24], and ultimately stimulates the differentiation of osteoclasts. The ERK, JNK, and p38 subfamilies are the main MAPK subfamilies. The binding of RANKL to RANK activates ERK through a series of reactions. ERK regulates the transcription of C-FOS after translocation to the nucleus, ultimately transforming mature macrophages into precursor osteoclasts [25]. Phosphorylated JNK activates AP-1 to promote the expression of MMP and ALP genes and stimulates the differentiation, survival, fusion, activation, and maturation of osteoclasts [26]. After the binding of RANKL to RANK, MEK6 phosphorylation is promoted and p38 is activated. Activated p38 is transferred from the cytoplasm to the nucleus, phosphorylating the transcription factor MITF and other proteins, ultimately promoting osteoclast differentiation [27]. In our study, PCA reduced the phosphorylation of ERK, JNK, and p38 in RAW264.7 cells treated with RANKL. The downregulation of MAPK expression induced by PCA was consistent with previously described results [28]. These results suggest that PCA may affect the fusion of precursor cells into osteoclasts by activating MAPK to suppress the expression of downstream factors.

NF-*κ*B signaling is another indispensable pathway in osteoclast induction [29]. The trimer of RANK-RANKL-TRAF6 activates NF-*κ*B. Then, NF-*κ*B separates from I-*κ*B and is quickly transported into the nucleus, binding to the promoters of the corresponding target genes and regulating osteoclast differentiation, maturation, and apoptosis [30, 31]. In the present study, PCA reduced the level of phosphorylated p65 in RANKL-induced osteoclasts. PCA suppressed RANKL-mediated osteoclast formation by inhibiting NF-*κ*B activity. PCA possibly inhibits the transcription of NFATc1 by restraining the phosphorylation of NF-*κ*B p65, thereby affecting the expression of downstream genes.

PCA is a water-soluble component of SM. SM and its other active ingredients are known to possess antiosteoporosis properties. Tanshinone is one of the most much-studied active components at present. Published studies have shown that tanshinone inhibits osteoclast activation and reduces bone absorption by destroying F-actin rings [32]. Cryptotanshinone also inhibits the formation of osteoclasts [33]. In our study, PCA reduced the number of TRAP-positive osteoclasts and the area of absorption pits, which proved that PCA inhibited the maturation and function of osteoclasts, suggesting that PCA has the potential to prevent bone loss and treat osteoporosis. Based on the findings of the present study, PCA exerts a synergistic effect with the abovementioned components of SM. This result further suggests that SM may also be an antiosteoporotic treatment that inhibits the maturation and function of osteoclasts.

Although some results were reported in our study, many other issues remain to be further explored. For example, how does PCA suppress the activation of MAPK and NF-*κ*B? Does PCA bind to cognate receptors on the cell surface of precursor cells and subsequently inhibit cellular signaling pathways that lead to NF-*κ*B and MAPK activation, or does PCA freely enter cells and directly inhibit NF-*κ*B and MAPK activation? Other questions include the effectiveness of PCA *in vivo* and its pharmacokinetics, which all require further study.

In conclusion, our research shows that PCA suppresses osteoclast differentiation by inhibiting MAPK and NF-*κ*B activation. Therefore, PCA potentially represents a cost-effective and alternative medicine for osteoporosis.

## Figures and Tables

**Figure 1:** PCA attenuates osteoclast differentiation induced by RANKL. (a) Viability of RAW264.7 cells exposed to PCA at different time points. (b) Viability of BMM cells exposed to PCA. (c) BMMs were induced to osteoclasts in 4 days. (d) Number of osteoclasts per well. (e) RAW264.7 cells were induced to differentiate into osteoclasts after 5 days. (f) Number of osteoclasts per well. (g) PCA (5 *μ*g/ml) was added to BMMs at three periods during the differentiation of osteoclasts. (h) Number of osteoclasts per well. A light microscope was used to acquire photomicrographs (magnification 10 × 10). Cells that were TRAP-positive and had more than three nuclei were considered osteoclasts. The quantities are presented as the mean ± SEM values (*n* = 3). ^∗^*P* < 0.01 and ^#^*P* < 0.05 compared with the control group.

**Figure 2:** PCA reduced bone absorption. (a) BMMs were grown in Osteo Assay Surface plates for 4 days (magnification 4 × 10). (b) Absorption area per well. (c) RAW264.7 cells were grown in Osteo Assay Surface plates for 7–8 days (magnification 10 × 10). (d) Resorption area per well. (e) TRAP staining of osteoclasts differentiated from BMMs on Corning CaP-coated plates (magnification 10 × 10). (f) Number of osteoclast per well. (g) Analysis of the absorption area per osteoclast-like cell. Absorption pits were quantified using ImageJ software. ^∗^*P* < 0.01 and ^#^*P* < 0.05 compared with the group treated with RANKL alone.

**Figure 3:** PCA reduces the size of F-actin rings. (a) A fluorescence microscope was used to capture the fluorescence images of F-actin rings (magnification 40x). (b) The F-actin ring size was quantified. ^∗^*P* < 0.01 compared with the M-CSF+RANKL group. (c) Flow cytometry was used to detect cells. (d) The ratios of apoptotic cells to control cells. ^∗^*P* < 0.01 compared with the control group.

**Figure 4:** PCA inhibits mRNA expression in RANKL-stimulated osteoclasts. ^∗^*P* < 0.01 compared with the RANKL group.

**Figure 5:** PCA suppresses the activation of the MAPK pathway. (a) Western blots showing protein levels. (b) The relative protein levels were compared with those in the group treated with RANKL alone. ^∗^*P* < 0.01 and ^#^*P* < 0.05 compared with the RANKL group.

**Figure 6:** PCA prevents RANKL-induced NF-*κ*B activation. (a) Western blots showing the levels of p-p65 and p65. (b) The protein levels were compared with those in the RANKL group. ^∗^*P* < 0.01 and ^#^*P* < 0.05 compared with the group treated with RANKL alone.

**Table 1:** The conditions and primer sequences used for RT-PCR.

Target genes	Primer sequences	Tm	Size
GAPDH	F: AGGTCGGTGTGAACGGATTTG	60	95
	R: GGGGTCGTTGATGGCAACA		

CTSK	F: CTCGGCGTTTAATTTGGGAGA	60	164
	R: TCGAGAGGGAGGTATTCTGAGT		

NFATc1	F: GGAGAGTCCGAGAATCGAGAT	60	102
	R: TTGCAGCTAGGAAGTACGTCT		

C-FOS	F: CGGGTTTCAACGCCGACTA	60	165
	R: TGGCACTAGAGACGGACAGAT		

MMP-9	F: GCAGAGGCATACTTGTACCG	60	229
	R: TGATGTTATGATGGTCCCACTTG		

DC-STAMP	F: GGGGACTTATGTGTTTCCACG	60	72
	R: ACAAAGCAACAGACTCCCAAAT		

## Data Availability

The datasets used and/or analyzed during the current study are available from the corresponding author on reasonable request.
